# Intelligent Recognition of Hospital Image Based on Deep Learning: The Relationship between Adaptive Behavior and Family Function in Children with ADHD

**DOI:** 10.1155/2021/4874545

**Published:** 2021-06-04

**Authors:** Hongyi Zhao, Jiangyu Chen, Yiqi Lin

**Affiliations:** ^1^Tianshui First People's Hospital, Tianshui 741000, China; ^2^The Second Affiliated Hospital and Yuying Children's Hospital of Wenzhou Medical University, Wenzhou 325000, China

## Abstract

Chronic diseases are gradually becoming the main threat to human health. By designing an efficient hospital management platform to quickly identify the corresponding chronic diseases, it can effectively reduce the labor cost, improve the accuracy of disease identification, and improve treatment efficiency. ADHD is a common behavioral disorder in school-age children, and it is also one of the most common chronic health problems in this period. The internationally recognized prevalence of ADHD is 3%–9%. ADHD often brings adverse effects on children's life and studying and at the same time increases difficulties for their families. Therefore, this paper designs an intelligent management platform for public hospitals based on a deep learning algorithm, evaluates the current situation and influencing factors of ADHD children through the child adaptive behavior scale and the family function assessment scale, and designs its intelligent platform by using a new technology of fNIRS. According to the nonlinearity and unsteadiness of the fNIRS signal, this paper proposes a motion noise removal method based on EMD algorithm methods: to automatically identify children with ADHD and improve the cognitive function of children with ADHD by intervention technology. The data are from the outpatients of the Department of Child Psychology of the First People's Hospital of Tianshui City in Gansu Province in 2018. The results showed that there were significant differences in the adaptive behavior scale (CABS) and fad scores between the two groups. In the seven dimensions of family function, there were significant differences between the two groups (*P* < 0.01). fNIRS management platform can effectively identify ADHD patients with high recognition accuracy. The intelligent management platform can significantly reduce the number of physical examination personnel, prolong the diagnosis and treatment time, reduce a lot of repetitive work, and improve the efficiency of diagnosis and treatment. At the same time, this technology also provides great help for better research and improvement of ADHD patients and provides a reference for the information intelligent construction of modern hospitals.

## 1. Introduction

Childhood ADHD is a typical behavior disorder of school-age children, and it is also one of the most common chronic health problems. They usually show obvious difficulty in concentration, short attention duration, and hyperactivity. It is not age-appropriate. More impulsive adult children will also affect their personal development, cause problems in daily work and life, interpersonal communication, and other aspects, and are more likely to become irritable, insecure, depressed, and even depressed. In addition, children are prone to drug abuse in adulthood, and the risk of antisocial personality disorder and behavior disorder is much higher than that of normal children. The risk of persistent emotional and destructive behavior disorder will also increase. Studying and mastering the image recognition method of ADHD patients based on deep learning has a positive impact on improving the problem behavior of ADHD children.

Many children with ADHD perform poorly at school, disobey their parents and teachers, disrupt the classroom, feel tired at school, and disobey because of symptoms. Their classmates will also exclude them, and their interpersonal relationships will be in trouble. It will also bring a lot of trouble and burden to the family. The relationship between parents and children is the most important type of relationship in the family. The disharmony between parents and children can lead to the development of ADHD children's bad behavior. The path can affect children's behavior through direct influence, such as the demonstration effect of parents' behavior, and indirect influence, such as the method of raising children or the interaction between parents and children.

The incidence rate of ADHD is increasing every year, which not only has a negative impact on children's physical and mental health but also has an overall impact on the overall quality of the nation and the future development of the country, which has brought many adverse effects to families, schools, and society. Green *J L* studied the association of ADHD spectrum disorder symptoms with social function, mental health, quality of life, and sleep in children with and without ADHD. ADHD was assessed through community-based screening and case confirmation using the child IV diagnostic interview schedule. Social interaction questionnaire was used to identify ASD symptoms, but there was no specific data [1]. Gonzalez Carpio *g* believes that traditional research studies on ADHD in children and adolescents mainly focus on the genetic and neurobiological aspects of the disease, but the role of family relationship has not been systematically studied. There is increasing evidence that the quality of parent relationship is correlated with ADHD symptoms in children. However, there is a lack of necessary experimental data [2]. Weyers *l* believes that the parallel phenomenon found in the study of attachment and attention deficit hyperactivity disorder indicates that there is a connection between the two structures. However, several articles on this tie have investigated all children with a possible expression of ADHD but have not found enough evidence to prove the link between ADHD and attachment. This study attempts to gather evidence that there may be a link between two aspects of ADHD in children with inattention. However, in the study of the impact of attachment on the disease, ADHD as a whole construction is not clear. Contrary to previous studies, only considering the types of inattention can completely alleviate this relationship by externalizing behavior problems. It is better to analyze it in the longitudinal study, but it lacks the content of numerical analysis [3]. Franke *s* said the study assessed possible correlations between behavioral profiles, quality of life and perceptions of social support, and parenting styles adopted by 26 mothers of children and adolescents with ADHD diagnosed by the same neurologist. The pattern characterized by negative behavior is related to the higher frequency of behavior problems and is related to the decrease of caregivers' adaptive function index, but some discussions are not accurate [4].

The innovation of this paper is to master the behavior and family situation of ADHD patients based on the evaluation scale. Using fNIRS, a new technology to establish a hospital intelligent management platform accurately identifies ADHD patients, intervenes ADHD children's families, comprehensively and deeply understands the parent-child relationship problems faced by ADHD children and their families, and explores ways to solve the problems. Through fNIRS technology, we can better master the information of patients, reduce the cost of human resources, and accelerate the construction of hospital automation. It has a positive effect on improving the diagnosis mode of disease.

## 2. Image Recognition Based on Deep Learning

### 2.1. Deep Learning

Deep learning is a new direction in the field of machine learning. Its main purpose is to create a processing mechanism similar to the human brain. A neural network simulates the human brain for analysis and data processing (such as image, text, sound, etc.) [5, 6]. The artificial neural network is a multilayer perceptron with many hidden layers [7]. The “depth” of deep learning refers to the number of layers of the neural network: the more the layers, the greater the depth of the network. Generally, the number of network layers is proportional to the ability to adapt to its functions. The traditional artificial neural network usually contains only one hidden layer, so its expression ability is limited [8, 9]. In order to improve the ability of the neural network to respond to complex functions, the network model constructed by deep learning is usually a deep neural network with multiple hidden layers. The model has a large number of parameters that can be trained. It has a stronger expression and learning ability [4]. As a method of studying features, deep learning actually uses some simple nonlinear models to transform the original features of data into more abstract and advanced expressions [2]. For the classification task, the high-level expression of data can usually enhance its classification ability and eliminate the influence of unnecessary factors [10]. The subsequent layer reorganization consists of the top-level research part to obtain the final abstract form of the target expression to be detected, as shown in Figure 1.

### 2.2. Multilayer Feedforward Network

#### 2.2.1. Perceptron Unit

The artificial neural network is composed of a large number of interconnected neurons [11, 12]. Among them, the neuron is the main module of the whole neural network. The neuron contains *n* inputs and one output. The formula for calculating source data is

(1) $$\begin{array}{c} \text{output}=f\left(h^{T}x+a\right)=\left(\sum_{i=1}^{n}h_{i}x_{i}+a\right), \end{array}$$

where *x* = (*x*_1_, *x*_2_,…, *x*_*i*_) is the input data, *h* = (*h*_1_, *h*_2_…, *h*_*i*_) is the network weight, *a* is the bias, and *f* () is the nonlinear activation function [13]. The input data is processed by a series of weighted summation and nonlinear activation functions to obtain the final result of neurons [13, 14]. The function of the nonlinear activation function is to realize nonlinear mapping between input data and output value.

#### 2.2.2. Multilayer Direct Transmission Network

The artificial neural network model is composed of the input layer, hidden layer, and output layer. The early artificial neural network is also called multilayer perceptron, *x* = (*x*_1_*x*_2_…, *x*_*i*_). *h*_*ji*_^*a*^ represents the weight parameter between the *i*th neuron of layer *a* and the *j*th neuron of layer *a* + 1. *r*_*j*_^*a*^ represents the results of the activation value of the output of the *j*th neuron in the network layer *a* which are as follows:

(2) $$\begin{array}{c} \overset{\left(2\right)}{\underset{1}{r}}=f\left(\overset{\left(1\right)}{\underset{11}{h}}x_{1}+\cdots \overset{\left(1\right)}{\underset{1n}{h}}x_{n}+\overset{\left(1\right)}{\underset{1}{a}}\right), \end{array}$$

(3) $$\begin{array}{c} \overset{\left(2\right)}{\underset{2}{r}}=f\left(\overset{\left(1\right)}{\underset{21}{h}}x_{1}+\cdots \overset{\left(1\right)}{\underset{2n}{h}}x_{n}+\overset{\left(1\right)}{\underset{2}{a}}\right). \end{array}$$

*s*_*a*_ is the number of neurons in the hidden layer of layer *a* as follows.

Because, in neural networks, the initial value of the hidden layer activation is usually used as the output of the next layer, the input value of the activation function of the *j*th neuron in layer *a* is the same as that in layer *a*:

(4) $$\begin{array}{c} \overset{a}{\underset{j}{c}}=\sum_{i=1}^{r_{a-1}}\overset{a-1}{\underset{ji}{h}}\overset{a-1}{\underset{i}{r}}+\overset{a-1}{\underset{j}{a}}. \end{array}$$

Input data is *x* = (*x*_1__,_*x*_2_…*x*_*i*__)_. After that, the forward propagation process of the multilayer feed-forward network is analyzed.

#### 2.2.3. Backpropagation Algorithm

The backpropagation algorithm is usually used in the process of training artificial neural networks [15, 16]. The main idea of the BP algorithm is to first calculate the error between the original value and the actual value of the neural network and then use the gradient descent algorithm to minimize the error function to continuously adjust and optimize the network parameters [17, 18]. Firstly, the loss function of a sample (*x*, *y*) is determined as follows:

(5) $$\begin{array}{c} J\left(h,a;x,y\right)=\frac{1}{2}{\left|f_{h,a}\left(x\right)-y\right|}^{2}, \end{array}$$

where *h* and *a* are the weight parameters of the network, which is a sample *f*_*h*,*a*_(*x*). The original value *y* obtained from the direct propagation of the network is the actual value corresponding to the sample *X*, {(*x*^(1)^, *y*^(1)^,…, *x*^(*m*)^, *y*^(*m*)^), *M* is the number of samples).

(6) $$\begin{array}{c} J\left(h,a\right)=\left[\frac{1}{m}\sum_{i=1}^{m}J\left(h,a;x^{i},y^{i}\right)\right]+\frac{\lambda }{2}{\left|\left|h\right|\right|}^{2}, \end{array}$$

(7) $$\begin{array}{c} \overset{a}{\underset{\text{new}}{c}}=c^{a}-\alpha \frac{\partial }{\partial c^{a}}J\left(h,c\right), \end{array}$$

where it is called the learning rate or step size factor, where the partial derivative is calculated as follows:

(8) $$\begin{array}{c} \frac{\partial }{\partial h^{a}}J\left(h,c\right)=\left[\frac{1}{m}\sum_{i=1}^{m}\frac{\partial }{\partial h^{a}}J\left(h,c;x^{\left(i\right)},y^{\left(i\right)}\right)\right]+\lambda h^{\left(a\right)}. \end{array}$$

### 2.3. Image Recognition

Image recognition is to recognize and classify the research objects according to their characteristics [19, 20]. For example, to identify 10 numbers written on cards from 0 to 9 to determine the size of the numbers on each card, this type of identification usually occurs in people's daily life. However, with the expansion and deepening of practice, the categories of things that people need to define become more and more complex, and the contents become more and more complex. In particular, with the improvement of science and technology, we can use the corresponding technology to transform the recognized objects into images or a series of data, namely, graphics and digitization. [21, 22]. But to recognize a pattern (whether it is data or image), extract its features, and then classify the features, the image recognition system shall include the following parts, and the system block diagram is shown in Figure 2:

The first part is to get the information about the image. The second part is image preprocessing. The preprocessing process includes the use of appropriate technical means to eliminate the noise and distortion of the original image, weaken the irrelevant features, and enhance the recognition system's more concerned function. If there are multiple recognition targets in the original image, it is necessary to use image segmentation technology to segment the original image into multiple images containing only one recognition target. The third part is the removal of objects. In order to ensure the accuracy of recognition, according to the predeveloped extraction principle, the features that have a greater impact on classification and recognition are selected.

### 2.4. Fuzzy Image Set Recognition Method

In fact, it is impossible to understand and analyze all problems only through clear boundaries. Fuzzy theory is introduced here to imitate human thinking. The process of identifying the method can be summarized as follows: calculate the degree of belonging of the sample to a specific category, that is, the degree of belonging to complete the model classification. The method of identifying template fuzzy sets can be simplified to the method of identifying the principle of maximum membership degree and the closest method of identifying the principle according to different principles.

#### 2.4.1. Recognition of Maximum Membership Principle

Let *f* be the domain of the object to be identified, *H*_1_*H*_2_⌃…*H*_*n*_ is an n-dimensional fuzzy set on *f*, and *f*_0_ ∈ *F* is an identified object element, if any:

(9) $$\begin{array}{c} H_{i}\left(f_{0}\right)=\max\left\{H_{k}\left(f_{0}\right)\right\}. \end{array}$$

#### 2.4.2. Approach Principle Recognition Method

In practical application, it may be found that the object to be identified is a fuzzy subset contained in universe *h*, and the expected pattern is also a fuzzy subset contained in universe H. In this case, special treatment is needed: let *B* and *C* be two fuzzy sets in the universe *H*, and *H* = (*f*_1_, *f*_2_,_…_*f*_*n*_) is a finite set definition:

(10) $$\begin{array}{c} M\left(B,C\right)={\left[\frac{1}{n}\sum_{i=1}^{n}\left|B\left(f_{i}\right)-C\left(f_{i}\right)\right|\right]}^{r\left(1/r\right)}. \end{array}$$

*R* is a positive real number. Let *m* (*B*, *c*) be the relative Minkowski distance of fuzzy sets *B* and *C*. If *r* = 1, then

(11) $$\begin{array}{c} M_{h}\left(B,C\right)=\frac{1}{n}\sum_{i=1}^{n}\left|B\left(f_{i}\right)-C\left(f_{i}\right)\right|. \end{array}$$

If *P*=22, then *M* (*B*, *c*) is called relative Euclid distance:

(12) $$\begin{array}{c} M_{E}\left(B,C\right)=\sqrt{\frac{1}{n}\sum_{i=1}^{n}\left|B\left(f_{i}\right)-C\left(f_{i}\right)\right|}. \end{array}$$

Let *n* fuzzy sets on universe *h*, *R* (*C*, *b*) be some closeness degree of fuzzy sets *C* and *B*, if there is *I* such that

(13) $$\begin{array}{c} R\left(C,B_{i0}\right)=\max\left\{R\left(C,B_{k}\right)\right\}. \end{array}$$

## 3. Investigation of Image Recognition in Children with ADHD

### 3.1. Etiology and Influencing Factors of ADHD in Children

The etiology and influencing factors of ADHD are mainly divided into three aspects: genetic factors, perinatal status and family, and psychological and social factors.

#### 3.1.1. Genetic Factors

Genetic factors are the key and important factors in the whole etiology. If the parents of children have different degrees of physical defects, chromosome abnormalities, mental disorders, etc., they will affect the children's brain development to varying degrees, resulting in hyperactivity.

#### 3.1.2. Perinatal Situation

If the mother of a child has abnormal reactions during pregnancy, premature delivery, or even poor nutrition, it will increase the prevalence of ADHD.

#### 3.1.3. Family, Psychological, and Social Factors

Family, psychological, and social factors play a very important role in ADHD. Family is the first environment for children's growth or life. What kind of mentality they have and what kind of interests they have all come from the influence of family.

### 3.2. Children's Adaptive Behavior Rating Scale

From January 2018 to October 2018, 200 children with ADHD aged 3–12 years were investigated. 178 valid questionnaires were collected, with an effective recovery rate of 89%. In the experimental group, there were 100 cases in total, and 93 cases received the effective questionnaire, with an effective recovery rate of 93%. All the patients were diagnosed by child psychiatrists through outpatient consultation, scale evaluation, behavior observation, nervous system examination, and other auxiliary examinations, and the generalized developmental disorder, mental retardation, and other major mental diseases were excluded. In the control group, 100 children aged 3–12 were selected from other departments in the same period, excluding mental diseases such as ADHD, nervous system diseases, mental retardation, physical diseases, learning difficulties, and emotional disorders. Finally, 85 valid questionnaires were collected, and the effective recovery rate was 85%. The survey plan was reviewed and approved by the ethics committee of the First People's Hospital of Tianshui city. The questionnaire survey of all subjects was carried out with the informed consent of their guardians, and the questionnaire was filled in by their guardians. The age and gender distribution of ADHD in children showed that ADHD was more common in children aged 6–9. Among them, 28 cases were 3–5 years old, accounting for 30.11%; 46 cases were 6–9 years old, accounting for 49.46%; 79 cases were male, accounting for 84.95%; and 14 cases were female, accounting for 15.05%. The results are shown in Table 1:

From the score of CABS, the score of the control group was higher than that of ADHD children. The difference in scores of the other six dimensions and 4 factors was statistically significant except for the difference in sensory movement and spatial-temporal trend between the two groups by *t*-test, as shown in Table 2.

### 3.3. Family Function Assessment Scale

The family environment is an important environment for children with ADHD to grow up in, and it is also an important factor leading to or aggravating ADHD symptoms. The relationship between family members, interaction, behavior thoughts and attitudes, and cultural literacy has little effect on the employment and growth of ADHD children. Only by establishing a harmonious and equal relationship between parents and children can we optimize the family environment and alleviate the symptoms of ADHD children. On the positive side, try more appropriate ways to raise children and give them more care and support. The scale contains some descriptions of families. Please read each project carefully and base on the last two months. Among the four possible answers, circle the number that best describes your family. For this reason, the survey scores are shown in Table 3:

### 3.4. Data Survey Summary Method

The independent function factor score, cognitive function factor score, social self-control factor score, and adaptive ability quotient (ADQ) in ADHD children's adaptive behavior scale were taken as the dependent variables, respectively, and the scores of 7 dimensions of the family function scale were 7 independent variables, and four multivariate regression models were constructed. The results are shown in Table 4. The four models were statistically significant (*P* < 0.01), and the *R* value of the complex correlation coefficient was between 0.341 and 0.669. Among them, the self-control factor and adaptive quotient factor are dependent variable models, which are statistically significant with the partial regression coefficient of three dimensions of family function.

### 3.5. Design of Intelligent Management Platform

The intelligent management platform is made according to the situation and quantity of children with ADHD. The system should provide the flexibility of operation as much as possible under the guidance of users. Authority management is an important guarantee of system flexibility; a user-friendly interface should fully reflect the people-oriented design concept and create a relaxed and pleasant experience for office users; try to use the simplest working method to realize the most powerful function, so as to provide a convenient system update and expansion according to the development requirements of measurement business. The successful operation of the system ensures a high exchange of measurement data, improves the scalability and maintainability of the system, and facilitates the collection and reading of the required situation and quantity of children with ADHD. fNIRS, as a noninvasive optical brain imaging technology, is very suitable for young children and other groups by virtue of its advantages of high ecological efficiency, portability, and long-time collection. It successfully describes the attenuation of light intensity as the function of the concentration of color cluster, molar extinction coefficient, differential path factor, and light source-detector distance, such as

(14) $$\begin{array}{c} OD\left(f,\lambda \right)=-\log\frac{H\left(f,\lambda \right)}{H_{0}\left(f,\lambda \right)}. \end{array}$$

## 4. Analysis of ADHD Patients and Intelligent Management Platform

### 4.1. Assessment and Analysis of Children's Adaptive Behavior

Through the comprehensive analysis and judgment of the rehabilitation of ADHD children, it is found that, in general, the rehabilitation of ADHD children is based on drug treatment. However, through a lot of practice and experience analysis, it is found that ADHD children are still faced with complex factors in the process of treatment, which are related to medical, social, psychological, ethical, and other aspects. With the continuous improvement of social work mechanisms and working methods, social work is becoming more and more important, more and more attention has been paid to the importance of work, and its role in solving the problems of children with ADHD is also playing an increasingly important role. The in-depth development and comprehensive application of social work children with ADHD are mainly characterized by lack of attention to affairs, low level of understanding of things, and lagging development of language and movement. In graduate school, they left places where they socialized, walked, or fought in class, and they did not have clear goals. In physical education class, these hyperactive children have poor body coordination and awkward posture. According to the questionnaire, the scores of children's ADHD adaptive behavior, such as sensory motor, are shown in Figure 3.

It can be seen from Table 3 that although the score in sensory movement is still very high, there are still many problems in the overall score. Compared with children of the same age, these hyperactive children have a superficial understanding of the problem, lower ability to judge things, and less control of the brain over the limbs, which leads to the children's involuntary excessive activities and the actions they carry out and practice. For example, relatively subtle forms of movement and the ability to flexibly control the body are not strong. The overall score of the questionnaire is shown in Figure 4.

Figure 4 shows that there is no absolute relationship between attention deficit hyperactivity disorder and brain behavior problems in children. These children usually do not have intellectual problems, but they have abnormal behavior, no specific reason is found, but the brain has a cerebellum. There is no definite conclusion about concussion. They often show that they cannot control their behavior and speak out loud in relatively quiet situations. They did not coordinate well during the movement. Although they are active, most of them are involuntary. In the process of movement, the limbs show movement and posture. It is very incongruous.

ADHD children's family function problems are more common, which will directly affect the formation of harmonious family relationships between parents and children. The relationship between parents and children is not only the earliest social relationship in the process of children's growth but also the most important relationship in the family relationship. Communication is all the communication between parents and children. Through these communication behaviors, all the information such as cognition, attitude, and emotion between parents and children can be transferred to each other. This survey scale contains some descriptions of families. The family function assessment scale is shown in Figure 5.

It can be seen from Table 4 that family has a great influence on children, and a bad parent-child relationship will affect the personality development of children with ADHD. If parents often ignore their children, regardless of their children, it is easy for them to form a selfish and indifferent character; children's personality needs to be positive and cheerful; parents of children with ADHD often lose faith, patience, etc. in their study guidance and life education due to the symptoms of hyperactivity and take simple and rude ways such as beating and scolding, which is easy to cause children to suffer. They are more likely to play truant, fight, and indulge in games and other behavioral problems, which is not conducive to the health of children.

### 4.2. Identification of ADHD Children Based on fNIRS Intelligent Software

ADHD usually occurs in childhood and often lasts until adolescence or even adulthood. About 5–8% of school-age children suffer from ADHD. These children with ADHD are difficult to control their own behavior or maintain attention, which has a very negative impact on their academic performance and social function. This disease increases the risk of other diseases, even if they are not directly associated with ADHD. Therefore, it is very important to explore an effective biological index for early diagnosis and intervention. In order to recognize ADHD children based on brain activity measured by fNIRS, we applied the hemodynamic response amplitude of the n-back task to the MVPA method. The signals collected by fNIRS do not fully represent brain functional activities and are often polluted by physiological system noise and the head movement-induced motion noise. Before the subsequent statistical analysis, these noises must be regressed. fNIRS is not so sensitive to motion noise, but head movement will still cause disturbance of fNIRS signals, such as sharp wave or baseline drift. A variety of methods have been developed to reduce the impact of motion noise, and then signal processing methods are used to detect and remove the motion noise, as shown in Table 5.

It can be seen from Table 5 that the effect of multichannel linear regression and ICA in removing motion noise is better, and when there is motion noise interference, HbO and Hb will become a positive correlation. By maximizing the negative correlation between HbO and Hb, the sharp wave will be removed, and the signal-to-noise ratio of the signal will be improved. Cooper et al. compared these methods and found that they achieved good results in their data. The relative concentrations of oxyhemoglobin and deoxyhemoglobin were measured by a near-infrared brain functional quantitative imaging system. Family changes such as family discord will be worse for children patients, such as 7–9 cm ms of EEG nerve potential and 6–10 mm of brain PET glucose and oxygen metabolism in children patients. A 3 × 11 measuring plate symmetrically covered the prefrontal and temporal lobes. There are 17 transmitters and 16 receivers alternately arranged on this measuring board, forming 52 measuring channels. The system adopts a 10 Hz sampling rate, as shown in Figure 6.

After preprocessing the fNIRS data, we calculated the average hemodynamic response of each channel of each subject under 1-back condition. The average value of each channel was taken as the feature extracted from each subject, based on the multivariable relationship between brain activity and behavior data. The higher the accuracy of the task, the faster the reaction, and the stronger the brain activity in the brain area. There is a correlation between brain activity and behavior data of the two groups under each condition. The error bar represents the 95% confidence interval of the bootstrap ratio. Based on multivariate pattern analysis, ADHD children and healthy control children were distinguished with very high classification accuracy, as shown in Figure 7.

In the fNIRS system, the common optical receiver probes include photomultiplier, photodiode, and avalanche photodiode. PMT is very sensitive to light, but it is limited to large volume, is sensitive to the magnetic field, and cannot be exposed to ambient light. PD has a high dynamic range, small volume, fast reaction speed, and no magnetic field sensitivity and can be exposed to ambient light. But because there is no amplifier in PD, it is necessary to design a low noise amplifier circuit to amplify the PD signal. APD has advantages similar to PD. In addition, the hemodynamic response patterns of the brain located in the lateral prefrontal lobe, middle and lower part of the prefrontal lobe, the right posterior prefrontal lobe, and the right temporal lobe have a strong ability to distinguish. The recognition pathway, especially the right lateral frontal lobe, is shown in Figure 8.

## 5. Conclusion

This paper studies the time spent between ADHD children, parents, and children. It is a key person in early childhood education and development, and the parent-child interaction model also has some impact on the future path of interpersonal interaction, because once the behavior pattern of ADHD children is formed, it is difficult to change. Therefore, it is more important for ADHD children to maintain or promote a good parent-child interaction model. However, the existing research results show that the pressure and interaction between parents and children in ADHD families are not optimistic. Therefore, rapid identification of chronic diseases is of great significance for the intelligent construction of medical institutions and the exploration of a good parent-child interaction model between ADHD children and their parents. In this paper, the behavior and family status of ADHD children were investigated by questionnaire, and the current situation of ADHD children was studied by specific experiments. According to the questionnaire survey, most ADHD children have the above defects in their behavior and family status. I hope to inspire parents of other autistic children and to enhance their understanding of special education professionals, social workers, and children. The public should understand the real situation of family interaction, and ADHD children should provide appropriate support from now on.

The scores of the dimensions of the Adaptive Behavior Scale (CABS) in children with ADHD and normal children were obtained by a two-sample *t*-test. The scores of language development, self-care, personal orientation, social responsibility, social self-control factor, labor skills, economic life, independent function, and cognitive function were all less than 0.01. The results showed that there were significant differences in the scores of ADHD children and normal children, and the scores of several dimensions of ADHD children were higher than those of ADHD children. Among them, the adaptive quotient of normal children was 108.06, and the adaptive quotient of children was 92.63, indicating that the adaptive ability of normal children was significantly higher than that of ADHD children. A study on the related factors of ADHD children in 2017 showed that there were significant differences between the ADHD group and control group in seven dimensions: sensory movement, self-care, personal orientation, social responsibility, social self-control factor, independent function factor, and ADQ (*P* < 0.01). Interestingly, no significant difference in sensorimotor dimension was found between the two groups. This study is aimed at children in Western China. At present, domestic ADHD research is mostly concentrated in the developed areas of Eastern China. The analysis results show that there are differences in influencing factors of ADHD among children in eastern and western China, and differences in geographical culture and family education concepts are the reasons for these differences. Among them, the personal orientation dimension and ADHD showed the strongest negative correlation.

This study first compares the children with ADHD and the normal children with the critical value of the family function by analyzing the scores of two groups of children on the family function scale (FAD). And then we analyze the critical value of the family function score between the children with ADHD and the normal children and evaluate their family function.

The results showed that the scores of six dimensions of family functional health in children with ADHD were higher than the critical value, indicating that family function in children with ADHD was in an unhealthy state in six dimensions of problem-solving, communication, role, emotional response, emotional intervention, and behavior control, while the scores of six dimensions of family functional health in normal children group were not above the critical value, but in a relatively healthy state. Meanwhile, the children with ADHD and normal children scored in each dimension of family function by a two-sample *t*-test. The results showed that there were significant differences in all dimensions of family functional health between the two groups except sensory movement and temporal and spatial orientation (*P* < 0.05). The family functional status of children in the normal group was better than that of children with ADHD, especially in the three dimensions of emotional response, emotional intervention, and behavioral control.

Based on the deep learning algorithm, an intelligent disease recognition algorithm is designed, which has good international adaptability and scientificity [23]. Foreign scholars have done relevant research on the use of big data in the field of medicine [24]. The virtual reality technology based on the Internet of things is prospective and practical [25]. Of course, highly developed hospital automation construction also needs to pay attention to medical data security [26].

The sample size of the study is small, and the sample size of ADHD girls is small. The difference between boys and girls in ADHD children's adaptive behavior is large, and the adverse relationship caused by feedback to the family is also different. The number of samples will be expanded in future research, and the weight of influencing factors between different genders will be more accurately determined.

## Figures and Tables

**Figure 1:** Deep learning process image (http://alturl.com/9p8rh).

**Figure 2:** Image recognition system.

**Figure 3:** Children's adaptive behavior outcome scale.

**Figure 4:** Children's adaptive behavior assessment survey.

**Figure 5:** Draw line chart for family function assessment.

**Figure 6:** The fNIRS probe is projected onto the brain mode.

**Figure 7:** Recognition accuracy of fNIRS.

**Figure 8:** Brain hemodynamic response pattern.

**Table 1:** Comparison of baseline data between ADHD group and normal control group.

variables	Cases (constituent ratio%)		*t/χ* ^*2*^	*P* value
	ADHD group (*n* = 93)	Control group (*n* = 85)		
*Gender*				
Male	79 (84.95%)	65 (76.47%)	2.065	0.151
Female	14 (15.05%)	20 (23.53%)		

*Age*				
Three–five	28 (30.11%)	35 (41.18%)	5.092	0.078
Six–nine	46 (49.46%)	42 (49.41%)		
Ten–twelve	19 (20.43%)	8 (9.41%)		
The average of age	7.19 ± 2.52	6.96 ± 2.35	0.626	0.532

**Table 2:** Comparison of CABS between the ADHD group and normal control group (mean ± SD).

Dimension	ADHD group (*n* = 93)	Control group (*n* = 85)	*T* value	*P* value
Sensorimotor	21.37 ± 2.68	20.94 ± 3.78	0.869	0.386
Life self-care	31.76 ± 9.42	36.39 ± 5.43	−3.964	≤0.001
Language ability	19.90 ± 6.29	25.47 ± 7.93	−5.211	≤0.001
Personal orientation	20.6 ± 5.07	31.25 ± 5.77	−13.099	≤0.001
Social responsibility	14.96 ± 3.76	20.73 ± 3.56	−10.499	≤0.001
Space-time	5.22 ± 3.41	5.26 ± 3.09	−0.089	0.929
Labor skills	4.16 ± 3.33	9.34 ± 4.90	−8.309	≤0.001
Economic activity	5.31 ± 3.20	7.38 ± 3.55	−4.078	≤0.001
Independent function factor	62.60 ± 16.16	74.05 ± 12.38	−5.267	≤0.001
Cognitive function factor	25.12 ± 9.34	30.73 ± 10.11	−3.849	≤0.001
Social/self-direction factor	35.56 ± 7.73	51.98 ± 8.12	−13.815	≤0.001
Adaptability quotient (ADQ)	92.63 ± 13.79	108.06 ± 11.84	−7.972	≤0.001

**Table 3:** Comparison of FAD between the ADHD group and normal control group (mean ± SD).

Dimension	Norms	ADHD group (*n* = 93)	Control group (*n* = 85)	*T* value	*P* value
Problem solving	2.20	2.23 ± 0.42	2.01 ± 0.37	3.66	≤0.001
Communication	2.20	2.23 ± 0.27	2.05 ± 0.25	4.66	≤0.001
Role	2.30	2.45 ± 0.31	2.25 ± 0.33	4.13	≤0.001
Emotional response	2.20	2.47 ± 0.28	1.95 ± 0.36	10.94	≤0.001
Emotional intervention	2.10	2.53 ± 0.51	2.30 ± 0.44	3.28	≤0.001
Behavior control	1.90	2.50 ± 0.32	1.85 ± 0.28	14.13	0.001
Total function	2.00	2.45 ± 0.21	1.92 ± 0.22	16.75	0.035

**Table 4:** Multiple linear regression analysis of FAD dimensions with CABS in the ADHD group (*n* = 93).

Independent variable	Independent function factor		Cognitive function factor		Social self-control factor		Adaptability value	
	*B*	*t*	*B*	*t*	*B*	*t*	*B*	*t*
Problem solving (*X*1)	−0.757	−0.227	−0.620	−0.290	−0.236	−0.122	−0.743	−0.250
Communication (*X*2)	−4.943	−0.947	−8.141	−2.428	−4.721	−1.558	−8.204	−2.242
Role (*X*3)	−3.556	−0.712	−2.096	−0.653	−0.242	−0.083	0.561	0.126
Emotional response (*X*4)	0.598	0.135	−3.269	−1.149	−2.050	−0.798	0.837	0.212
Emotional intervention (*X*5)	−3.394	−0.908	0.396	0.165	−5.944^∗^	−2.739	−4.486	−1.345
Behavior control (*X*6)	−7.749	−1.647	−7.74^∗^	−2.563	−10.339	−3.788	−11.902	−2.837
Total function (*X*7)	−11.606^∗^	−1.984	−5.302	−1.412	−13.753	−4.053	−14.128	−2.708
*F*	3.186^*∗∗*^		3.798^*∗∗*^		19.664^*∗∗*^		7.904^*∗∗*^	
*R*	0.341		0.368		0.669		0.496	

*B* is the regression coefficient, and *T* is the hypothesis test value of the corresponding regression coefficient.

**Table 5:** Characteristics of brain imaging techniques.

Type	Measurement	Information	Time resolution	Portability	Cost
fNIRS	HbO and Hb	4∼6 cm	Per second	Yes	Medium
fMRI	BOLD	5 mm	Per second	No	High
EEG	Nerve potential	7∼9 cm	Millisecond	No	High
PET	Glucose and oxygen metabolism	6∼10 mm	About 60 seconds	No	High

## Data Availability

The data cannot be shared without permission from the data provider.
